The article "Game Analysis on the Influence of Participants' Psychology on Value Co-Creation in Community E-Commerce Platform Supply Chain" was published in 2022. Journal: Comput Intell Neurosci.

# Game Analysis on the Influence of Participants' Psychology on Value Co-Creation in Community E-Commerce Platform Supply Chain

**DOI:** 10.1155/2022/4684068

**Published:** 2022-07-14

**Authors:** Liu Ziyu, Zhao Lixia

**Affiliations:** School of Economics and Management, Hebei University of Science and Technology, Shijiazhuang, China

## Abstract

As e-commerce continues to develop, online shopping is becoming more and more popular, and community e-commerce platform emerges as the times require. To make the participants in the supply chain of community e-commerce platform play a greater role in value creation, the supply chain of community e-commerce platform can get more benefits. This paper studies the psychology of all participants in the supply chain of community e-commerce platform, so as to establish the value creation mechanism of community e-commerce platform. Through the research, it is found that by studying the psychology of the two main participants in the supply chain of community-based online store, community e-commerce platform and community leader, and considering whether they will do their best to participate in value co-creation, a two-party evolutionary game model is constructed. By calculating the dynamic replication equation, the influence of the psychology of the participants in the supply chain of the community-based online store on the supply chain revenue of the community-based online store is obtained, and the evolutionary trend of both parties in the game is simulated by Matlab. It is concluded that the key factors that affect the co-creation of the value of a community-based online store supply chain are the proportion of increased income, the cost of participating in co-creation of value, and the purchasing power of consumers brought by participating with both parties. Finally, some suggestions and countermeasures are put forward through the analysis of simulation results.

## 1. Introduction

With the development of e-commerce, more and more retail models have gradually emerged, and community group buying, live delivery and big data have become hot words. Community e-commerce group buying such as Youxuan, Kuaituan, TaoCaicai came into being. At the end of 2018, community group buying developed rapidly in second-and third-tier cities, becoming one of the hottest investment tracks. Due to the imperfection of community group purchase, when the community-based online store was initially developed, the community-based online store frequently exploded. At the beginning of 2020, there was a major public health incident in novel coronavirus all over the world. Under the epidemic situation, students could not attend classes normally and staff could not get to work on time, which had a great impact on people's lives. The epidemic situation inevitably had an impact on people's daily life and China's development, and how people could purchase their daily life and supply their daily necessities became an urgent problem. In this case, some traditional industries have been greatly impacted, and even many enterprises have closed down. On the contrary, it is precisely in this special case that the network service industry has shown strong development potential, and many community platforms have emerged as the times require. For example, the supply chain of community-based online stores such as Meituan Optimization and Buy More Food has begun to enter our field of vision widely, which has provided convenience for our life under the epidemic situation, not only reduced the close contact between people, but also made farmers' backlog of goods under the influence of the epidemic situation.

The article "Game Analysis on the Influence of Participants' Psychology on Value Co-Creation in Community E-Commerce Platform Supply Chain" was published in 2022. Journal: Comput Intell Neurosci.

The mode of “prepurchase + self-delivery” in community group purchase means that the merchants presell the goods first, then uniformly deliver the goods from the local warehouse or different producing areas, and finally let the community customers self-deliver the goods. The group purchase mode can not only effectively control the quality of the goods, but also achieve centralized purchasing on demand and has high cost performance. It directly skips the logistics cost and management cost caused by stocking, reduces the transportation and storage time of the goods, ensures the freshness of the goods to the greatest extent, reduces the loss, and reasonably solves the problem of after-sales of the goods [1]. If the quality of the goods received by consumers is problematic or different from expectations, they only need to contact the head of the delegation to solve the after-sales problem. How to maximize the value of a community-based online store, and in the supply chain of community platform, what is the impact of the psychology of community leaders and community e-commerce platform on the co-creation of value of community-based online store supply chain? How to maintain the stability of value creation? By studying the game of community-based online store supply chain co-creation of value, this paper concludes that whether the psychology of community leaders and community e-commerce platform tries their best has a great influence on community e-commerce platform co-creation of value, and the community leaders get benefits through the commission of community e-commerce platform and the commission of consumers' purchasing power, which solves how to maintain the stability of community-based online store platform supply chain co-creation of value.

The article "Game Analysis on the Influence of Participants' Psychology on Value Co-Creation in Community E-Commerce Platform Supply Chain" was published in 2022. Journal: Comput Intell Neurosci.

American scholar C.K. Prahalad clearly put forward the word “co-creation of value,” which holds that enterprises can jointly create value by using the capabilities and resources of their business partners, suppliers and customers, thus winning the competition in the market [2]. This behavior can be described by dialogue, acquisition, risk management and transparency, that is, DART framework [3]. In terms of supply chain co-creation of value, the output of many enterprises is not only pure commodities, but also services to customers, so some scholars have made relevant research on service supply chain co-creation of value. Gao et al. [4] first proposed the co-creation of value mechanism of logistics service supply chain under the service-oriented logic, and also introduced the main content of the service-oriented logic in this paper. The service-oriented logic pointed out that the obvious transformation in economy is not only the transformation from goods to services, but also the transformation of resources from tangible to intangible and from static to dynamic. Later, Zhao and Chen [5] reviewed the Logistics Serve Supply Chain (LSSC) and service-oriented logic, studied the influence of interaction and integration on LSSC co-creation of value, then divided and combined them according to different dimensions, and discussed the influence of interaction and integration on LSSC co-creation of value from three aspects. They are resource integration under tactical interaction, relationship integration under strategic interaction and network integration under operational interaction, which are the important influencing factors of LSSC co-creation of value. With the development and operation of the logistics service supply chain in enterprises, to maintain the stable operation of the logistics service supply chain in enterprises, Lu [6] established a two-party game model of how to realize co-creation of value between customer enterprises and integrated logistics enterprises in the logistics service supply chain by using evolutionary game, analyzed the evolutionary game process and simulated it with Python, so as to obtain the key factors affecting the value trend of the logistics service supply chain. The results show that the integration mechanism and interaction mechanism jointly realize the co-creation of value process of logistics service supply chain, and at the same time, we should pay attention to the position and role of customer enterprises in co-creation of value.

Other scholars have also studied the co-creation of value of e-commerce platform. Under the O2O(Online To Offline) business model, Chen [7] studied the mature retail industry in O_2_O business ecosystem from the perspective of the evolution of O_2_O business ecosystem, analyzed the composition system of business ecosystem and the realization process of multi-co-creation of value, and revealed the realization mechanism of multi-co-creation of value in retail industry in O_2_O business ecosystem. Under the C2M (Customer To Manufacturer) business model, Liu and Wang [8] took C2M e-commerce platform as the research object, analyzed the process of C2M e-commerce platform co-creation of value, analyzed each stage of C2M e-commerce platform co-creation of value activities, and combined with some related cases, put forward the upgrading and evolution mechanism of C2M e-commerce platform, and divided the C2M e-commerce platform co-creation of value system into three types, namely unbalanced, ecological community and bilateral. Li et al. [9] studied the modes of cross-border e-commerce. There are mainly B2B (Business To Business) and B2C (Business To Customer) modes of cross-border e-commerce, and digital empowerment plays an important role in the process of realizing co-creation of value. Through the article research, it is found that in the product selection stage, manufacturing and purchasing stage and sales stage of cross-border e-commerce, Digital technology plays an all-round role in empowerment, and digital empowerment can effectively promote the co-creation of value process of cross-border e-commerce, thus realizing the interaction and integration of resources under digital empowerment. Wang et al. [10] studied the trust crisis of e-commerce platform, proposed a consumer-to-business-to-consumer model based on margin policy for e-commerce platform, and gave three modes under margin policy based on two-way game: unit price trading mode, double price trading mode and consumer reporting behavior mode, the revenue of e-commerce platform can be maximized. Wu et al. [11] found that there is no stable equilibrium point in the model through modeling, theoretical derivation and analysis, and concluded that increasing the cooperative income and commission coefficient can encourage the government to adopt supervision strategies, and allowing consumers to take part in supervision can make e-commerce platforms make better decisions, by this way, the value of e-commerce platform can be maximized. From the perspectives of co-creation of value [12], process components [13] and IT service projects [14], scholars have studied e-commerce and given corresponding suggestions.

The article "Game Analysis on the Influence of Participants' Psychology on Value Co-Creation in Community E-Commerce Platform Supply Chain" was published in 2022. Journal: Comput Intell Neurosci.

From the above literature, we can see that at present, there are few literature on the comprehensive study of community-based online store platform supply chain co-creation of value. By studying the psychological relationship between participants and participants in community-based online store platform supply chain, this paper first clarifies the composition and operation process of community-based online store platform supply chain. Secondly, the evolutionary game model between community-based online store platform and community leader is established by evolutionary game method. This paper explores the influence of community-based online store platform and community leader psychology on co-creation of value in community-based online store platform supply chain by considering the factors such as whether the participants' psychology try their best to take part in the cost of co-creation of value, the proportion of community-based online store platform supply chain increasing revenue when the participants' psychology try their best, and the psychology of main consumers in community-based online store platform supply chain that affects both parties' revenue. This paper makes up for the research gap of community-based online store platform supply chain co-creation of value, and also lays some foundations for future scholars to study community-based online store platform. As consumers are the important subjects of community-based online store platform co-creation of value, this paper studies community-based online store platform co-creation of value by considering consumers' psychology, and establishes a co-creation of value mechanism, so that community e-commerce platform supply chain can get better benefits.

## 2. Composition of Community-Based Online Store Platform Supply Chain Value Co-Creation

The community-based online store platform supply chain refers to the relationship between suppliers and consumers established by the community-based online store platform, taking the needs of consumers as the starting point, integrating all resources in the chain, so as to realize the links of supply, production, circulation and consumption, and combining the business needs of every participant in the community-based online store platform supply chain, making the links of supply, sorting and distribution closely cooperate and seamlessly link, so as to maximize the overall interests and value creation of the community-based online store platform supply chain. According to the actual situation, participants in the supply chain of community-based online store platform can be divided into suppliers, community-based online store platforms, grid station service providers, community leaders and consumers.

1. Suppliers. The supply chain of community-based online store platform is different from our usual supply chain of convenience stores and supermarkets. Their suppliers are not only simple wholesalers, but also many online fruits and vegetables. Their suppliers are manufacturers and farmers. They can join in as suppliers through the platform and directly supply commodities to the supply chain of community-based online store platform, which is why many commodities of community-based online store platform are cheaper than offline ones.
2. community-based online store platform. The community-based online store platform displays the goods provided by suppliers on the platform, where consumers can buy and buy goods, and when there is a problem with the goods, they can apply for refund in small programs or clients. The community-based online store platform also has a head end, where the head can handle the orders of consumers in time. The community-based online store platform is a bridge between suppliers and consumers, suppliers and heads, heads and consumers. Community leaders. When registering, the community leader can set the position of the pick-up point by himself, and can contact the delivery master to urge the goods. In addition, in the supply chain of community-based online store platform, the community leader plays the role of providing after-sales service to consumers. If there is a problem with the products, consumers only need to contact the leader to deal with it, and after the leader's approval, the platform will refund the corresponding money to consumers. Head of delegation is the bridge between community-based online store platform and consumers.
3. Grid station service providers. The grid station service providers are transit stations of the warehouse and self-pick-up point in the city center. The requirements for the grid station service providers are as follows: there are places for storing goods, vehicles for delivery, receiving and delivery personnel, etc. The grid service providers are not only the distributor of the supply chain of the community-based online store platform, but also need to undertake the sorting business of the community-based online store platform, and be responsible for delivering the goods purchased by consumers to the offline delegation leaders' self-raising point on time to ensure the quality. Grid service providers play a vital role in the supply chain of the whole community-based online store platform.
4. Community leaders. When registering, the community leaders can set the position of the pick-up point by himself, and can contact the delivery master to urge the goods. In addition, in the supply chain of community-based online store platform, the community leaders play the role of providing after-sales service to consumers. If there is a problem with the products, consumers only need to contact the leaders to deal with it, and after the leaders' approval, the platform will refund the corresponding money to consumers. Head of delegation is the bridge between community-based online store platform and consumers.
5. Consumers. Consumers have a high degree of participation in the whole community-based online store platform supply chain sales process. They browse and select the products provided by suppliers on the community-based online store platform, and then buy the products they need. Products with good user experience can also be recommended to consumers in the whole community in the community commodity exchange group, while products with bad experience can also be fed back to the head of the delegation in the community commodity exchange group.

The article "Game Analysis on the Influence of Participants' Psychology on Value Co-Creation in Community E-Commerce Platform Supply Chain" was published in 2022. Journal: Comput Intell Neurosci.

Through the analysis of the supply chain main body of community-based online store platform, the relationship among several participants in the supply chain of community-based online store platform is shown in Figure 1.

## 3. Community-Based Online Store Platform Supply Chain Value Co-Creation Evolution Game Model Construction

### 3.1. Applicability of Evolutionary Game Theory in Value Co-Creation of Community-Based Online Store Platform Supply Chain

In the traditional game, it is generally believed that the psychology of the participants in the game is completely rational, and the participants make the game under the condition of complete information. However, in real economic life, it is difficult to realize the participants' complete rationality and complete information. In each enterprise's cooperation and competition, each participant's psychology is different. In Evolutionary Game Theory, people are no longer modeled as super-rational players, but they think that people can achieve game equilibrium by trial and error for many times. Finally, the equilibrium selected by trial and error for many times is a function of achieving the equilibrium process, so the individual benefits of participants and some or some details in the whole equilibrium process will have an impact on the equilibrium of the game. The process of co-creation of value, interaction and integration of participants in the supply chain of community-based online store platform cannot completely realize the co-creation of value of the whole supply chain at a certain moment. It is difficult for the managers of participants or participants themselves to be completely rational when facing complex problems, and many complicated related factors need to be considered. Then, through trial-and-error step by step, it is possible to achieve a certain degree of optimal decision-making. The psychology of each participant also needs repeated coordination, so as to cooperate with each other to achieve a stable cooperative and competitive relationship. Only then can community leaders, grid station service providers and community-based online store platform gradually gain their highest value in the supply chain, and at the same time, they can help other participants realize value, so as to achieve value creation and benefit sharing. Therefore, it is reasonable and realistic to use evolutionary game to study the influence of psychology among participants in the supply chain of community-based online store platform on co-creation of value.

The article "Game Analysis on the Influence of Participants' Psychology on Value Co-Creation in Community E-Commerce Platform Supply Chain" was published in 2022. Journal: Comput Intell Neurosci.

### 3.2. Parameter Setting of Game and Establishment of Profit Matrix

#### 3.2.1. Basic Assumptions

Community-based online store platform supply chain participants' roles in the whole supply chain co-creation of value and their roles are also different. Suppliers supply the platform by joining the community-based online store platform, and the community-based online store platform is delivered to the community leader through grid station service providers, so that consumers can pick up the goods at the pick-up points set by the community leader, thus completing the whole process of the community-based online store platform supply chain. However, due to some differences between the interests of community leaders and community-based online store platform, the psychological uncertainty of community-based online store platform managers and community leaders for the whole supply chain and the different strategies of both parties to obtain revenue, the following two assumptions are made.

**Hypothesis 1 .**

Participants. Assume that the two actors involved in the evolutionary game are the community leader of the supply chain of the community-based online store platform and the community-based online store platform. The influencing factor is consumers. The community-based online store platform sends goods to the community leader's pick-up point through the grid station service provider, while consumers can pick them up at the community leader's pick-up point by placing orders on the e-commerce platform. The purchasing power of consumers determines the commission of community leaders and the benefits of community-based online store platform.

**Hypothesis 2 .**

Psychological hypothesis. Due to the profit-seeking nature of the participants in the supply chain of community-based online store platform, community-based online store platform and community leaders may not try their best to take part in co-creation of value in the process of co-creation of value, so the game strategy set is to try their best to take part in co-creation of value and not try their best to take part in co-creation of value.

1. Community-based online store platform and community leaders do their best to take part in co-creation of value. By consulting the community leader and calling the community-based online store platform for telephone consultation, it can be concluded that if both parties will do their best to take part in co-creation of value, they will do the following:
2. First of all, the preferential treatment of community goods. The community-based online store platform will do its best to carry out preferential activities on the platform and strictly manage the community leaders, and at the same time, the leaders will vigorously publicize the preferential activities in the community exchange group. Then, the interaction between community-based online store platform and community leaders. The community-based online store platform should also set some numerical values. When the number of orders placed by community members under the community leader reaches the numerical value, the commission percentage of the community leader should be increased. By changing the commission for the community leaders through the community-based online store platform, the community leaders can be encouraged to participate more fully in value creation. At the same time, the community leaders also need to constantly feedback the favorable comments and negative comments of community members to the community-based online store platform when increasing the commission, and remind the community-based online store platform to make corresponding improvements, so as to improve the benefits of the community-based online store platform. Finally, integrate the information of community members and evaluate all orders, so as to achieve better co-creation of value. According to the number of orders placed by members of different communities for the same commodity and the frequency of orders placed by members of the same community for the same commodity on different dates, we can know the feedback of commodities. The community-based online store platform can choose to continue purchasing the corresponding commodities, and the community leader should share the statistical information with members of the community in time, so as to promote the better sales of these commodities.
3. Community-based online store platform and community leaders did not fully take part in co-creation of value. Although the community leaders have joined the community-based online store platform, the community leaders may not take his duties seriously, such as publicizing the products of the community-based online store platform and timely handling the return orders of community members. However, the community-based online store platform does not give the community leaders appropriate preferential policies, and also choose to turn a blind eye to the feedback and suggestions of the community leaders, which lead to the decline in the sales of commodities on the community-based online store platform and the poor experience of community members on the community-based online store platform, which lead to the lack of trust between the two parties, mutual blame, insufficient efforts and conscientious efforts to promote the sales of commodities, and thus lead to a decline in the profits of both parties.

The article "Game Analysis on the Influence of Participants' Psychology on Value Co-Creation in Community E-Commerce Platform Supply Chain" was published in 2022. Journal: Comput Intell Neurosci.

Assuming that the probability of community-based online store platform choosing to do its best to take part in co-creation of value of community-based online store platform supply chain is *x*, the probability of choosing not to do its best to take part in co-creation of value is 1 − *x*, where 1; The probability of community leaders choosing to do their best to take part in co-creation of value in the supply chain of community-based online store platform is *y*, and the probability of choosing not to do their best to take part in co-creation of value is 1 − *y*, where.

In the process of evolutionary game between community-based online store platform and community leader, the strategies that can be selected are (try their best to participate, not try their best to participate), and the strategies that partners can choose when participating in the business of platform enterprises are (try their best to participate, not try their best to participate). The game strategy combination of both sides is shown in Table 1.

#### 3.2.2. Parameter Setting

Through the co-creation of value analysis of community-based online store platform supply chain (see Table 2), the parameters are set as follows (see Table 3).

#### 3.2.3. Establishment of Income Matrix

As participants in the evolutionary game, community-based online store platform and community leader, community-based online store platform and community leader can get basic benefits in the community-based online store platform without choosing any publicity methods. When the community-based online store platform and community leaders begin to participate in value co-creation, the community leaders need to pay personal time, and the community-based online store platform needs to give preferential treatment to commodities. Although it has paid a certain cost, it has made contributions to the supply chain and achieved co-creation of value, and both parties can get more benefits. Therefore, the final income of both parties should be the income obtained without any publicity and preferential treatment plus the income obtained through co-creation of value, minus the cost paid in the process of co-creation of value.

The article "Game Analysis on the Influence of Participants' Psychology on Value Co-Creation in Community E-Commerce Platform Supply Chain" was published in 2022. Journal: Comput Intell Neurosci.

Based on the above analysis and previous basic assumptions, the payment matrix of the evolutionary game of co-creation of value between community-based online store platform and community leader in the supply chain of community-based online store platform can be constructed as shown in Table 4.

#### 3.2.4. Local Stability Analysis

(1) The benefits of community-based online store platform.
When the community-based online store platform chooses to fully take part in value co-creation, the benefits obtained by the community-based online store platform are as follows:
  (1) $$\begin{array}{c} U_{a1}=y\left(a+K_{a}\times \text{ef}-C_{\text{ab}}\right)+\left(1-y\right)\left(a-E_{b}\right). \end{array}$$
When the community-based online store platform chooses not to fully take part in value co-creation, the benefits obtained by the community-based online store platform are as follows:
  (2) $$\begin{array}{c} U_{a2}=y\left(a+\theta_{a}\times a-S_{\text{ab}}\right)+\left(1-y\right)\left(a-E_{b}+\theta_{a}\times a-S_{\text{ab}}\right). \end{array}$$
Therefore, the total revenue of community-based online store platform participating in value co-creation is:
  (3) $$\begin{array}{c} U_{a}={\text{xU}}_{a1}+\left(1-x\right)U_{a2}. \end{array}$$
Then the dynamic equation of community-based online store platform participating in value co-creation is:
  (4) $$\begin{array}{c} \frac{\text{d}x}{\text{d}t}=x\left(U_{a1}-U_{a}\right). \end{array}$$
Substitute formula (1) and (3) to get the dynamic equation:
  (5) $$\begin{array}{c} F_{X}\left(x\right)=\frac{\text{d}x}{\text{d}t}=x\left(1-x\right)\left[y\left(K_{a}\times \text{ef}-C_{\text{ab}}+\theta_{a}\times a+S_{\text{ab}}\right)+\left(1-y\right)\left(S_{\text{ab}}-\theta_{a}\times a\right)\right]. \end{array}$$
(2) Benefits of community leaders.
When the community leader chooses to fully take part in value co-creation, the benefits obtained by the community leader are as follows:
  (6) $$\begin{array}{c} U_{b1}=x\left(b+K_{b}\times \text{ef}-C_{\text{ba}};\right)+\left(1-x\right)\left(b+\theta_{b}\times b-S_{\text{ba}}\right). \end{array}$$
When the community leaders choose not to do his best to take part in value co-creation, the benefits obtained by the community leader are as follows:
  (7) $$\begin{array}{c} U_{b2}=x\left(b-E_{a}\right)+\left(1-x\right)\left(b-E_{a}+\theta_{b}\times b-S_{\text{ba}}\right). \end{array}$$
Therefore, the total benefits of community leaders' participation in value co-creation are:
  (8) $$\begin{array}{c} U_{b}={\text{yU}}_{b1}+\left(1-y\right)U_{b2}. \end{array}$$
Then the dynamic equation of community leaders' participation in co-creation of value is:
  (9) $$\begin{array}{c} \frac{\text{d}y}{\text{d}t}=y\left(U_{b1}-U_{b}\right). \end{array}$$
Substitute formula (6) and (8) to get the dynamic equation:
  (10) $$\begin{array}{c} F_{y}\left(y\right)=\frac{\text{d}y}{\text{d}t}=y\left(1-y\right)\left[x\left(K_{b}\times \text{ef}-C_{\text{ba}}+\theta_{b}\times b+S_{\text{ba}}\right)+\left(1-x\right)\left(S_{\text{ba}}-\theta_{b}\times b\right)\right]. \end{array}$$
(3) Equilibrium point analysis.
The participating community-based online store platform and community leaders of both sides will take part in the process of co-creation of value of the supply chain of the community-based online store platform while maximizing their interests. They will constantly change their strategies of participating in co-creation of value, so as to achieve the evolutionary stability strategy, and make formulas (5) and (10) equal to 0 respectively, that is:
  (11) $$\begin{array}{c} F_{X}\left(x\right)=\frac{\text{d}x}{\text{d}t}=x\left(1-x\right)\left[y\left(K_{a}\times \text{ef}-C_{\text{ab}}+\theta_{a}\times a+S_{\text{ab}}\right)+\left(1-y\right)\left(S_{\text{ab}}-\theta_{a}\times a\right)\right]=0,\\ F_{y}\left(y\right)=\frac{\text{d}y}{\text{d}t}=y\left(1-y\right)\left[x\left(K_{b}\times \text{ef}-C_{\text{ba}}+\theta_{b}\times b+S_{\text{ba}}\right)+\left(1-x\right)\left(S_{\text{ba}}-\theta_{b}\times b\right)\right]=0. \end{array}$$
Get *x* = 0, *x* = 1 and *y*^*∗*^=*θ*_*a*_*a* − *S*_ab_/*K*_*a*_ef − *C*_ab_; *y* = 0, *y* = 1 and *x*^*∗*^=*θ*_*b*_*b* − *S*_ba_/*K*_*b*_ef − *C*_ba_, five local equilibrium points of the system can be obtained: E1(0, 0), E2(0, 1), E3(1, 1), E4(1, 0), *E*5=(*θ*_*a*_*a* − *S*_ab_/*K*_*a*_ef − *C*_ab_, *θ*_*b*_*b* − *S*_ba_/*K*_*b*_ef − *C*_ba_)
The replication dynamic equation of community-based online store platform (5) can be obtained by taking partial derivative of *x*:
  (12) $$\begin{array}{c} \frac{\partial F_{x}\left(x\right)}{\partial x}=\left(1-2x\right)\left[y\left(K_{a}\times \text{ef}-C_{\text{ab}}+\theta_{a}\times a+S_{\text{ab}}\right)+\left(1-y\right)\left(S_{\text{ab}}-\theta_{a}\times a\right)\right]. \end{array}$$

**Situation 1 .**

The article "Game Analysis on the Influence of Participants' Psychology on Value Co-Creation in Community E-Commerce Platform Supply Chain" was published in 2022. Journal: Comput Intell Neurosci.

When *y*^*∗*^=*θ*_*a*_*a* − *S*_ab_/*K*_*a*_ef − *C*_ab_, The probability that the community leader chooses to try his best to participate is *θ*_*a*_*a* − *S*_ab_/*K*_*a*_ef − *C*_ab_, d*x*/d*t*  = 0 is forever established, If the duplicate dynamic equation is stable, then in the range of [0, 1], the stable solution of the dynamic equation is constant as *x*, and one of the critical values of the evolutionary game process is *x*.

**Situation 2 .**

When 0 < *y* < *θ*_*a*_*a* − *S*_ab_/*K*_*a*_ef − *C*_ab_ (0 < *θ*_*a*_*a* − *S*_ab_/*K*_*a*_ef − *C*_ab_ < 1, substitute 0, 1 into formula (13) to get *∂*d*x*/d*t*/*∂*(*x*=0) < 0, *∂*d*x*/d*t*/*∂*(*x*=1) > 0, according to the stability condition, it is known that *x* = 0 is a stable solution. When the probability of community leader B implementing reasonable participation strategy is less than, Therefore, no matter how the supply chain of community-based online store platform evolves, community-based online store platform A will not do its best to take part in co-creation of value, but will choose not to do its best to take part in co-creation of value at all. Finally, neither the community-based online store platform nor the community leader will do their best to take part in co-creation of value at the same time. At this time, the benefits of community-based online store platform not doing its best to take part in co-creation of value are greater than those of fully participating in co-creation of value. Because both parties involved in the evolutionary game are rational, in this case, the result of the game is that community-based online store platform tends not to do its best to take part in co-creation of value, and community leaders prefer not to do their best to take part in co-creation of value, so that both community-based online store platform and community leaders are not doing their best to take part in co-creation of value.

**Situation 3 .**

When *θ*_*a*_*a* − *S*_ab_/*K*_*a*_ef − *C*_ab_ < *y* < 1, substitute *x* = 0 and *x* = 1 into formula (13) to obtain, *∂*d*x*/d*t*/*∂*(*x*=0) > 0, *∂*d*x*/d*t*/*∂*(*x*=1) < 0, When *∂dx*/*dt*/*∂*(*x*=1) < 0, *x* = 1 is a stable solution, That is to say, When the community leader B chooses to do his best to take part in value co-creation and community-based online store platform, the probability is greater than *θ*_*a*_*a* − *S*_ab_/*K*_*a*_ef − *C*_ab_, After a long-term evolution in the supply chain of community-based online store platform, community-based online store platform will finally choose to do its best to take part in value co-creation. Because the benefit of community-based online store platform's full participation in community-based online store platform's supply chain value co-creation is greater than that of community-based online store platform's full participation in supply chain co-creation of value, both sides of evolutionary game will eventually choose to fully take part in co-creation of value.

For the community leader's replication dynamic equation (10) to get partial derivative of *y*, the explanation of the process result is similar.

The article "Game Analysis on the Influence of Participants' Psychology on Value Co-Creation in Community E-Commerce Platform Supply Chain" was published in 2022. Journal: Comput Intell Neurosci.

Through the above analysis and partial derivation, we can get the Jacobian matrix of the above game model as follows:

(13) $$\begin{array}{c} J=\left(\begin{array}{cc} \partial F\left(x\right)/\partial x & \partial F\left(x\right)/\partial y\\ \partial F\left(y\right)/\partial x & \partial F\left(y\right)/\partial y \end{array}\right). \end{array}$$

According to Jacobian matrix analysis: When the equilibrium point is (0, 0), The trace of Jacobian matrix is (*S*_*ab*_ − *θ*_*aa*_ − *θ*_*bb*_ + *S*_*ab*_).The sign of the trace is closely related to the setting of the initial value, so the trace is uncertain. The stability of the equilibrium point can be obtained by the local stability analysis of the Jacobian matrix obtained by this system [15]. The determinant of Jacobian matrix is (*S*_*ab*_ − *θ*_*aa*_) (*S*_*ab*_ − *θ*_*ab*_), When the set initial values are different, the results of Jacobian matrix will be different, so substituting into the equilibrium point cannot get the value of determinant or judge the symbol of trace.

## 4. Simulation Analysis of Community-Based Online Store Platform Supply Chain Co-Creation of Value

Based on the above analysis, the community e-commerce platform and the community leader may try their best to take part in the co-creation of value of the supply chain of the community e-commerce platform, or they may choose not to take part in the value co-creation of the supply chain of the community-based online store platform. The final result of the evolutionary game between the two parties will also be related with the setting of parameter values and the specific assignment, so the evolutionary model is simulated with Matlab. By changing the numerical value of each parameter, it simulates whether the community-based online store platform and the community leader do their best to take part in the co-creation of value process of the supply chain, and analyzes the influence of the change of the proportion (*K*_*i*_) that the participants do their best to increase profits in the supply chain of the community-based online store platform, the change of the cost (*C*_*ij*_) that the participants do their best to take part in co-creation of value and the change of consumers' purchasing power (*f*) that both participants do their best to take part in on the supply chain profits of the community-based online store platform. According to many experiments and investigations on the assignment of parameters, as shown in Table 5, assuming that the community-based online store platform of the community-based online store platform has no publicity and preferential treatment, the income a is 50, the commission *b* of the community leaders have no publicity and preferential treatment is 30, the extra unit income *e* obtained after both participants do their best to take part in co-creation of value and promote consumer purchasing power is 2, and the consumer purchasing power *F* brought by both participants is 10. The proportion Ka of community-based online store platform doing its best to increase revenue in the supply chain of community-based online store platform is 0.1, the proportion Kb of community leaders doing their best to take part in the supply chain of community-based online store platform is 0.4, the proportion *θ*_*a*_ of community-based online store platform not doing their best to take part in co-creation of value is 0.6, the proportion *θ*_*b*_ of community leaders not doing their best to take part in co-creation of value is 0.4, and the cost *C*_*ab*_ required by community e-commerce doing their best to take part in co-creation of value is 10. The cost *C*_*ba*_ required for community leaders to fully take part in co-creation of value is 8, the cost *S*_*ab*_ required for community-based online store platform not to fully take part in co-creation of value is 5, the cost *S*_*ba*_ required for community leaders not to fully take part in co-creation of value is 4, the impact *E*_*a*_ of community-based online store platform not to fully take part in co-creation of value on community leaders' income is 3, and the impact *E*_*b*_ of community leaders not to fully take part in co-creation of value on community-based online store platform's income is 5.

The article "Game Analysis on the Influence of Participants' Psychology on Value Co-Creation in Community E-Commerce Platform Supply Chain" was published in 2022. Journal: Comput Intell Neurosci.

### 4.1. Participants Try Their Best to Take Part in the Influence of the Change of the Ratio of Increasing Profits (*K*_*i*_) in the Supply Chain of Community-Based Online Store Platform on the Evolution Results

The community-based online store platform does its best to increase the profit ratio of the supply chain of the community-based online store platform. The influence of the change of *K*_*a*_ on the community-based online store platform and community leaders is shown in Figures 2 and 3.

When the community leaders do their best, the simulation results of the influence of the change of the proportion *K*_*b*_ of the supply chain of the community-based online store platform on the community-based online store platform and the community leaders are shown in Figures 4 and 5.

Through the analysis of the simulation diagram, it can be seen that the higher the *K*_*i*_ value of the participants' best participation in the community-based online store platform supply chain to increase revenue, the faster the participants choose to do their best to take part in the value co-creation of the community-based online store platform supply chain, which shows that the larger the proportion of participants' best participation in the community-based online store platform supply chain to increase revenue, the more willing both parties are to do their best to take part in the co-creation of value of the community-based online store platform supply chain.

The article "Game Analysis on the Influence of Participants' Psychology on Value Co-Creation in Community E-Commerce Platform Supply Chain" was published in 2022. Journal: Comput Intell Neurosci.

### 4.2. The Influence of the Change of the Cost (*C*_*ij*_) Required by the Participants to Do Their Best to Take Part in Co-creation of Value on the Evolution Results

The community-based online store platform does its best; the cost required by the supply chain of the community-based online store platform; the influence of the change of C_ab_ on the community-based online store platform and community leaders; the simulation results are shown in Figures 6 and 7.

When community leaders do their best to take part in co-creation of value, the simulation results of the influence of the change of *C*_*ba*_ on the community-based online store platform and community leaders are shown in Figures 8 and 9.

Through the analysis of the simulation diagram, it can be seen that when both parties choose to do their best to take part in the supply chain of community-based online store platform at a high level (greater than or equal to 30), the increase of the cost of community leader and community-based online store platform participating in the supply chain of community-based online store platform will lead to the result being biased towards *x* = 0 and *y* = 0, that is, both parties do not do their best to take part in co-creation of value, which shows that both parties participating in the evolutionary game should try their best to control the cost at a low level while participating in co-creation of value.

### 4.3. The Influence of the Changes of Consumers' Purchasing Power (*f*) Brought about by the Best Efforts of Both Participants on the Evolution Results

The simulation results of the influence of the change of consumer purchasing power *f* brought by the participation of both participants on the community-based online store platform and community leaders are shown in Figures 10 and 11.

Other parameters in the dynamic equation remain unchanged, making *f* equal to 10, 30 and 100, respectively, to get the simulation diagram. Through the analysis of the simulation diagram, we can see that the higher the purchasing power *f* of consumers brought by the full participation of both participants, the faster the two participants choose to fully take part in the value co-creation of the community-based online store platform supply chain, which shows that the higher purchasing power of community consumers will make the community-based online store platform and community leaders have more information and motivation to continue to take part in co-creation of value, and the cooperative relationship will be more stable, and both parties can also take part in the community more fully.

The article "Game Analysis on the Influence of Participants' Psychology on Value Co-Creation in Community E-Commerce Platform Supply Chain" was published in 2022. Journal: Comput Intell Neurosci.

## 5. Conclusions and Countermeasures

More and more community-based online store platforms are gradually coming into our field of vision, and the competition among them is increasing. They are composed of community leaders, community-based online store platforms, consumers, suppliers and grid station service providers. All participating entities take part in co-creation of value, and realize co-creation of value by integrating resources through interaction between the participating entities. This paper mainly studies whether the two main participants in the supply chain of the community-based online store platform, the community-based online store platform and the community leader, will do their best to take part in co-creation of value, constructs an evolutionary game model between the two parties, and obtains the main influencing factors of the supply chain income of the community-based online store platform by calculating the dynamic replication equation. Finally, the key factors are simulated by Matlab. The decision-making evolution trend of both parties participating in the supply chain game of community-based online store platform is simulated, and the corresponding countermeasures are put forward through the analysis of the simulation results, so as to improve the willingness of community leaders and community-based online store platforms to do their best to take part in co-creation of value.

The conclusions are as follows:

1. Only when the community-based online store platform and the community leader choose to do their best to take part in the co-creation of value of the community-based online store platform, the final benefit is greater than the final benefit of choosing not to do their best to take part in the co-creation of value of the supply chain of the community-based online store platform, will there be the possibility of combining the two strategies (do their best to participate, do their best to participate) and (do not do their best to participate).
2. Through the calculation of two-party evolutionary game model, it is concluded that the key factors are the proportion (*K*_*i*_) that participants do their best to take part in the supply chain of community-based online store platform to increase profits, the cost (*C*_*ij*_) that participants do their best to take part in co-creation of value and the purchasing power (*f*) of consumers brought by their full participation with both parties. Among them, the proportion (*K*_*i*_) that participants do their best to take part in the supply chain of community-based online store platform and the purchasing power of consumers (*f*) that both parties do their best to take part in promote the enthusiasm of co-creation of value, while the cost (*C*_*ij*_) that participants do their best to take part in co-creation of value inhibits the enthusiasm of co-creation of value.

The article "Game Analysis on the Influence of Participants' Psychology on Value Co-Creation in Community E-Commerce Platform Supply Chain" was published in 2022. Journal: Comput Intell Neurosci.

To improve the enthusiasm of community leaders and community-based online store platforms to take part in co-creation of value, the following suggestions are put forward for the supply chain of community-based online store platforms:

1. Increase customer purchasing power through community-based online store platforms' favoured efforts and community leaders' advertising. Consumers' pleasure with the community-based online shop platform determines their psychology, and consumers' psychology determines the entire income of the community-based online store platform's supply chain. Through activities such as spike killing, snapping up, and group buying, the community-based online store platform should improve consumers' trust and love psychology to the community-based online store platform, which not only improves the purchasing power of existing old consumers in the supply chain of the community-based online store platform, but also improves the purchasing power of new consumers in the supply chain of the community-based online store platform, however, it is also possible to publicize the community-based online store platform by increasing consumer goodwill towards the platform, resulting in more new users joining the platform, increasing the number of consumers, increasing the sales volume of the platform's products, and increasing the benefits of the community-based online store platform's supply chain. To improve consumers' experiences of the community-based online shop platform, community leaders should deal with community members' requests for after-sales processing in a timely manner. They should also aggressively share high-volume products with members of the community exchange group,
2. so as to increase the frequency of products appearing in consumers' sight. The high frequency and the feedback from other consumers in the group will drive more community members to place orders for products with high sales volume, thus forming a virtuous circle.
3. Improve the transparency of information, strengthen the trust between the community-based online store platform and community leaders, so as to motivate both parties to take part in value creation. The relevant policies and plans of the supply chain of the community-based online store platform should be announced in time, and the community leader should also feedback the feedback information of community members in the community exchange group to the community-based online store platform in time, so as to prompt the community-based online store platform to adjust suppliers and commodities in time, and the transparency of information will make both parties involved trust each other more, thus participating in value creation more actively.
4. Establish win-win psychology for both sides. Although the community-based online store platform and the community leader are two independent entities with their interests, the community leader hopes that the community-based online store platform can provide them with more commissions, while the community-based online store platform hopes that the community leader can create more benefits for the community-based online store platform with less commissions. Community leaders and community e-commerce platforms should establish a win-win mentality for both sides. However, if only egoism is the core, regardless of the interests of the partners, the gains of both parties will be reduced, so both the community e-commerce platform and the community leader should change their psychology, regard each other as a community of destiny, work together, share risks, and do their best to take part in the value creation of the supply chain of the community-based online store platform.

The article "Game Analysis on the Influence of Participants' Psychology on Value Co-Creation in Community E-Commerce Platform Supply Chain" was published in 2022. Journal: Comput Intell Neurosci.

The development of community-based online store platform supply chain has become a new supply chain model. When the epidemic happened, the community-based online store platform supply chain provided us with convenience, avoided close contact between people, delivered to the community, and solved the problem that people could not go out under the epidemic. Now the epidemic situation has improved, and the community-based online store platform supply chain has become a complete supply chain model. Through the research of this paper, the community-based online store platform supply chain is provided with participation, which makes the community-based online store platform supply chain provide a good management direction for the management participants. It also provides a guide for the state to supervise the community-based online store platform supply chain in the future, and also provides a foundation for scholars to study the community-based online store platform supply chain. The state should give support and open attitude to the community-based online store platform supply chain and develop a new supply chain model.

Finally, this paper only analyzes the whole industrial chain of the community-based online store platform supply chain, but for a community-based online store platform, we need to make a specific analysis of the specific enterprise, and introduce corresponding policies and management modes according to the development of the enterprise itself.

The article "Game Analysis on the Influence of Participants' Psychology on Value Co-Creation in Community E-Commerce Platform Supply Chain" was published in 2022. Journal: Comput Intell Neurosci.

## Figures and Tables

**Figure 1:** Schematic diagram of the relationship between supply chain participants of community-based online store platform.

**Figure 2:** When the community-based online store platform does its best, the proportion of the supply chain of the community-based online store platform increases revenue, and the influence of *K*_*a*_ change on the community-based online store platform simulation results.

**Figure 3:** When the community-based online store platform does its best, the proportion of the supply chain of the community-based online store platform increases revenue, and the influence of *K*_*a*_ change on the community leaders simulation results.

**Figure 4:** The proportion of community leaders' best efforts to increase revenue in the supply chain of community-based online store platform *K*_*b*_ change affects the community-based online store platform simulation results.

**Figure 5:** The community leaders' best efforts to increase the profit ratio of the supply chain of the community-based online store platform *K*_*b*_ changes influence the community leaders simulation results.

**Figure 6:** Simulation results of the influence of the change of the cost *C*_*ab*_ required by the supply chain of the community-based online store platform on the community-based online store platform when the community-based online store platform does its best.

**Figure 7:** Simulation results of the influence of the change of the cost *C*_*ab*_ required by the supply chain of the community-based online store platform on the community leader when the community-based online store platform does its best.

**Figure 8:** When community leaders do their best to take part in co-creation of value, the change of the cost *C*_*ba*_ required by the supply chain of community-based online store platform influences the simulation results on the community-based online store platform.

**Figure 9:** Simulation results of the influence of the change of *C*_*ba*_ on community leaders when community leaders try their best to take part in the co-creation of value of community-based online store platform supply chain.

**Figure 10:** Simulation results of the influence of the change of consumer purchasing power f brought by the participation of both participants on the community-based online store platform.

**Figure 11:** Simulation results of the influence of the change of consumers' purchasing power f caused by the participation of both participants on community leaders.

The article "Game Analysis on the Influence of Participants' Psychology on Value Co-Creation in Community E-Commerce Platform Supply Chain" was published in 2022. Journal: Comput Intell Neurosci.

**Table 1:** Game strategy combination between community-based online store platform and community leaders.

		Community leaders	
		Try their best to participate	Not try their best to participate
Community-based online store platform	Try their best to participate	(Try their best to participate, try their best to participate)	(Try their best to participate, not try their best to participate)
	Not try their best to participate	(Not try their best to participate, try their best to participate)	(Not try their best to participate, not try their best to participate)

**Table 2:** Influencing factors of value co-creation between community-based online store platform and community leaders.

Value co-creation	Behavior	Profit	Cost
Interaction mechanism	Share consumer order information	Get commission and income from consumers' orders.	Communication cost time cost
Integration mechanism	Relational integration, resource integration	Improve the popularity of platform and commodities, so as to obtain higher commissions and benefits.	Communication cost time cost

**Table 3:** Main parameters and their meanings.

Direct earnings	*a*	The benefits of community-based online store platform without any publicity and preferential treatment
	*b*	Commission for community leaders without any publicity or preferential treatment

Synergistic earnings	*e*	Both parties of the participants do their best to participate in value co-creation, and gain extra unit income after promoting the purchasing power of consumers
	*f*	Consumers' purchasing power brought by the participation of both parties to the main body
	*K*_*a*_	Community-based online store platform does its best to increase the proportion of revenue in the supply chain of community-based online store platform
	*K*_*b*_	Community leaders do their best to participate in the supply chain of community-based online store platform to increase the proportion of revenue
	*θ*_*a*_	The community-based online store platform does not do its best to participate in value co-creation to increase the revenue ratio
	*θ*_*b*_	Community leaders do not try their best to participate in value co-creation to increase the income ratio.

Cost	*C*_*ab*_	The community e-commerce will do its best to participate in the cost of value co-creation
	*C*_*ba*_	Community leaders do their best to participate in the cost of value co-creation
	*S*_*ab*_	The community-based online store platform does not try its best to participate in the cost of value co-creation
	*S*_*ba*_	The community leader does not do his best to participate in the cost of value co-creation
	*E*_*a*_	Community-based online store platform does not fully participate in the impact of value co-creation on the income of community leaders
	*E*_*b*_	The influence of community leaders' efforts to participate in value co-creation on the revenue of community-based online store platform

The article "Game Analysis on the Influence of Participants' Psychology on Value Co-Creation in Community E-Commerce Platform Supply Chain" was published in 2022. Journal: Comput Intell Neurosci.

**Table 4:** Benefit matrix of community-based online store platform and community head participating in co-creation of value.

		Community leaders	
		Do their best to participate *y*	Not do their best to participate1 − *y*
Community-based online store platform	Do his best to participate *x*	*a*+*K*_*a*_ × ef − *C*_ab_; *b*+*K*_*b*_ × ef − *C*_ba_;	*a* − *E*_*b*_; *b*+*θ*_*b*_ × *b* − *S*_ba_;
	Not do his best to participate 1 − *x*	*a*+*θ*_*a*_ × *a* − *S*_ab_; *b* − *E*_*a*_;	*a* − *E*_*b*_+*θ*_*a*_ × *a* − *S*_ab_; *b* − *E*_*a*_+*θ*_*b*_ × *b* − *S*_ba_;

**Table 5:** Initial parameter settings.

Parameters	*a*	*b*	*e*	*f*	*K*_*a*_	*K*_*b*_	*θ*_*a*_	*θ*_*b*_	*C*_*ab*_	*C*_*ba*_	*S*_*ab*_	*S*_*ba*_	*E*_*a*_	*E*_*b*_
Numerical value	50	30	2	10	0.1	0.4	0.6	0.4	10	8	5	4	3	5

## Data Availability

The data used to support the findings of this study are included within the article.
